This article has been retracted.

# Analysis of the Curative Effect and Prognostic Factors of Anterior Cervical Surgery for Spinal Cord Injury without Radiographic Abnormalities

**DOI:** 10.1155/2022/6836966

**Published:** 2022-08-08

**Authors:** Jian Tan, Fanchen Hu, Jun Ou, Xiaotao Su, Jingnan Liu

**Affiliations:** The Affiliated Nanhua Hospital, Department of Spinal Surgery, Hengyang Medical School, University of South China, Hengyang, Hunan 421000, China

## Abstract

**Objective:**

The study aimed to investigate the effect of anterior cervical surgery in the treatment of spinal cord injury without radiographic abnormalities (SCIWORAs) and analyze the related factors affecting the prognosis of patients.

**Methods:**

A total of 86 patients with SCIWORA who were admitted to our hospital from June 2018 to March 2021 were selected as the research subjects. According to the different treatment methods selected by the patients, they were divided into the control group (*n* = 38) and the observation group (*n* = 48). The control group was treated with conservative therapy, and the observation group was treated with anterior cervical total laminectomy decompression, internal fixation, and bone graft fusion. The efficacy of the treatment was assessed preoperatively and 6 months after surgery using the Japanese Orthopedics Association (JOA) functional evaluation criteria for cervical spinal cord injury. The improvement rate of the JOA score at the last follow-up visit was calculated according to the Hirabayashi formula to evaluate the prognosis of patients.

**Results:**

The JOA score of the observation group six months after surgery was (14.98 ± 2.75) that was higher than that of the control group (12.16 ± 2.54) (*P* < 0.05). After surgery, the improvement rate of the JOA score in the observation group was higher than that in the control group (*P* < 0.05). After surgery, the scores of health condition, physiological function, and role physical in the observation group were (23.18 ± 1.09), (22.75 ± 1.54), and (22.64 ± 1.46), which were higher than those in the control groups (20.94 ± 1.65), (20.26 ± 1.78), and (19.56 ± 1.82) (*P* < 0.05). The results of univariate analysis showed that the ASIA classification of cervical spinal cord injury, the type of MRI cervical spinal cord injury, the scope of cervical spinal cord injury, lumbar disc herniation, and the time from injury to treatment were all related to the prognosis of the patients (*P* < 0.05). Multivariate analysis showed that the ASIA classification of cervical spinal cord injury, the type of MRI cervical spinal cord injury, the scope of cervical spinal cord injury, and the time from injury to treatment were the independent factors affecting the prognosis of patients (*P* < 0.05).

**Conclusion:**

For patients with SCIWORA, anterior total lamina decompression and internal fixation with bone grafting and fusion can effectively promote the recovery of cervical spinal cord function and improve the prognosis and quality of life of patients. The ASIA classification of cervical spinal cord injury, the type of MRI cervical spinal cord injury, the scope of cervical spinal cord injury, and the time from injury to treatment were the independent prognostic factors for patients.

## 1. Introduction

Spinal cord injury without radiographic abnormalities (SCIWORAs) refer to the cervical spinal cord injury in which a patient has clinical symptoms of cervical spinal cord and nerve injury, but there is no imaging manifestation such as fracture and dislocation on X-ray and CT [1, 2]. Patients without fracture-dislocation type cervical spinal cord injury are not uncommon in clinic, and the incidence shows an increasing trend along with the aging of the population [3, 4]. SCIWORA is mostly caused by mild and moderate external forces, and clinical treatment is often divided into two ways, i.e., surgical treatment and conservative treatment. In the past, conservative treatments were mostly advocated, such as detumescence, inhibition of inflammatory response, nutritional nerve, and external fixation of the cervical vertebra [5, 6]. However, with the rapid development of medical technology and great progress of medical imaging technology in recent years, especially the extensive application of MRI technology, further research has beencarried out on the injury mechanism, clinical characteristics, treatment prognosis, and other aspects of the injury. For adult patients, most surgeons advocate surgical treatment in clinic at present [7, 8]. Anterior cervical decompression and bone grafting and internal fixation are the main surgical method for clinical treatment of adult SCIWORA, which can relieve the symptoms of cervical spinal cord compression and repair and reconstruct the cervical spine structure [9, 10]. The purpose of this study was to investigate the efficacy of anterior cervical surgery for SCIWORA and to analyze the related factors affecting the prognosis of patients.

## 2. Materials and Methods

### 2.1. Patients

A total of 86 patients with SCIWORA who were admitted to our hospital from June 2018 to March 2021 were selected as the research subjects. Inclusion criteria were as follows: according to the trauma history, clinical manifestations and signs of patients, combined with cervical X-ray or CT, and MR examination, SCIWORA was definitely diagnosed; patients with different degrees of clinical symptoms such as neck pain, limb pain, or numbness; all patients and their family members were explained the possible curative effects of surgical treatment and conservative treatment, and the patients or their family members chose the treatment independently. Exclusion criteria were as follows: patients with unstable vital signs; patients with severe craniocerebral and thoracic trauma; patients with psychiatric disorders; patients with poor response to conservative treatment were later converted to surgical treatment; patients were followed up during the process of shedding. According to the different treatment methods selected by the patients, they were divided into the control group (*n* = 38) and the observation group (*n* = 48). There was no significant difference in general data between the two groups (*P* > 0.05), as shown in Table 1.

### 2.2. Treatment Methods

The observation group was treated with anterior cervical total lamina decompression internal fixation and bone grafting fusion. The patient took the supine position with a soft pillow under the shoulder and a moderate backward extension of the head. According to the level of spinal cord injury or the spinal cord compression site of the patient, a transverse incision on the right side of the anterior neck was taken and the skin was cut. The subcutaneous tissues were separated layer by layer and entered along the muscular space until reaching the front of the vertebral body, where the responsible segments were fully exposed. According to the intraoperative X-ray results of the *C*-arm, the surgical segments were determined again, and the decompression range was determined again according to the preoperative CT or MR examination results of the cervical spine of the patient. If the lesion was a vertebral body, subtotal corpectomy bone graft fusion internal fixation was performed directly. If the lesion was an intervertebral disc, decompression bone graft fusion internal fixation was performed through the intervertebral disc. The posterior longitudinal ligament of the vertebral body is subjected to acute separation and resection, and for the posterior longitudinal ligament with adhesion or calcification, grinding can be performed first, followed by separation and resection. Subsequently, the patient's ilium was taken for bone grafting and fusion and fixed with the anterior cervical titanium plate. After surgery, all patients were administered dehydrating agents, low-dose glucocorticoids, neurotrophic drugs, infection prevention, and other general treatment. For patients who could move their limbs, they were instructed to carry out functional exercise as soon as possible, and especially for patients who could walk with their lower limbs, they were instructed to wear neck girth and other supports to move out of bed as soon as possible after removing the drainage tube.

Patients in the control group received comprehensive conservative treatment. Patients with trauma were treated with debridement, suture, and hemostasis, patients' vital signs were monitored, and patients were guided to stay in bed and rest quietly. Mannitol injection (Huaren Pharmaceutical (Rizhao) Co., LTD., National Drug Approval Word: H37021265) was administered at 250 g/time, 1 time/d, for intravenous infusion; 40 mg of methylprednisolone sodium succinate (Sinopagic Rongsheng Pharmaceutical Co., LTD., National Drug Approval Letter: H20030727) injection was added into 100 mL of 0.9% sodium chloride injection, once a day, for intravenous infusion. Then, 40 mg of monosialotetrahexose ganglioside sodium injection (Qilu Tianhe Huishi Pharmaceutical Co., LTD., National Drug Approval: H20056783) was added into 100 mL of 0.9% sodium chloride injection, once a day, for intravenous drip. Meanwhile, the blood pressure and blood glucose levels of the patients were controlled to be stable, the protection of gastric mucosa of the patients was strengthened, and nutritional intervention was strengthened. After 3 weeks of treatment, the patient's neck was fixed with a neck brace for 2 months.

### 2.3. Observation Indicators

#### 2.3.1. Cervical Spinal Cord Function

Preoperative and 6 months after operation, the patients were scored with the JOA spinal cord function score issued by the Japan Orthopedics Association [11]. The total score was 0∼17 points. The higher the score was, the better the spinal cord function would be.

#### 2.3.2. Determination of the Therapeutic Effect

The improvement rate of the JOA score at the last follow-up visit was calculated according to the Hirabayashi formula, and the improvement rate  = ((last follow-up score − score before surgery)/(17 − score before surgery)) × 100%. The improvement rate above 75% was considered as excellent, 50%∼74% as good, 25%∼49% as fair, and less than 25% as poor.

#### 2.3.3. Quality of Life Scoring

6 months after surgery, the patients' health condition, physiological function, role physical, and emotional function were scored using the Short Form Quality of Life Scale (SF-36) in four dimensions, with 0∼25 points for each dimension. A higher score indicated a higher quality of life.

#### 2.3.4. Prognosis

The prognosis of patients was evaluated according to the improvement rate of the JOA score, and the patients were divided into the excellent group and the poor group.

### 2.4. Statistical Methods

All data were processed with SPSS 22.0 statistical software. The enumeration data were examined by the *X*^2^ test and expressed by (*n* (%)), and the measurement data were examined by the *t*-test and expressed by ($\bar{x}\pm s$). Multivariate analysis adopted the multiple logistic regression model. The difference is statistically significant when *P* < 0.05.

## 3. Results

### 3.1. Comparison of Cervical Spinal Cord Function between the Two Groups

After the operation, the JOA score of the observation group (14.98 ± 2.75) was higher than that of the control group (12.16 ± 2.54) (*P* < 0.05) as shown in Figure 1.

### 3.2. Comparison of Efficacy between the Two Groups

After operation, there were 15 cases of excellent, 11 cases of good, 10 cases of fair, and 2 cases of poor in the control group, and the excellent and good rate was 68.42% (26/38). In the observation group, 26 cases were excellent, 16 cases were good, and 6 cases were fair, and the excellent and good rate was 87.50% (42/48). The excellent and good rate of the JOA score in the observation group (87.50%) was higher than that in the control group (68.42%) (*P* < 0.05) as shown in Figure 2.

### 3.3. Comparison of Patients' Quality of Life Scores between the Two Groups

After operation, the scores of health condition, physiological function and role physical in the observation group were (23.18 ± 1.09), (22.75 ± 1.54), and (22.64 ± 1.46), which were higher than those in the control group (20.94 ± 1.65), (20.26 ± 1.78), and (19.56 ± 1.82) (*P* < 0.05) as shown in Figure 3.

### 3.4. Univariate Analysis of Prognosis of Patients

The results of univariate analysis showed that the ASIA classification of cervical spinal cord injury, the type of MRI cervical spinal cord injury, the scope of cervical spinal cord injury, lumbar disc herniation, and the time from injury to treatment were all related to the prognosis of the patients (*P* < 0.05) as shown in Table 2.

### 3.5. Analysis of Multiple Factors Affecting Prognosis of Patients

Multivariate logistic analysis showed that the ASIA classification of cervical spinal cord injury, the type of MRI cervical spinal cord injury, the scope of cervical spinal cord injury, and the time from injury to treatment were the independent factors affecting the prognosis of patients (*P* < 0.05) as shown in Tables 3 and 4.

## 4. Discussion

When the cervical vertebra suffers from hyperextension force, the cervical spinal cord is squeezed by the intervertebral discs protruding from the front and the folds of the ligamentum flavum in the rear, resulting in the injury with the central tube of the cervical spinal cord as the center, and then, the hemorrhage and edema around the central tube are the main pathological changes; central necrosis of the spinal cord may occur in severe cases [12, 13]. The pathogenesis of SCIWORA is based on the existence of pathological factors in the spinal canal that reduces the reserve space, such as cervical disc herniation. These potential pathological factors or symptoms are mild and neglected. When acute violence causes cervical hyperextension or hyperflexion, the cervical spinal canal is acute narrowed, and the posterior yellow ligament buckling occurs, resulting in compression injury to the spinal cord [14, 15]. Before MRI examination is applied to the diagnosis of this disease, due to the lack of sufficient imaging data to support, conservative treatment is usually adopted. With the development and application of MRI, we can not only visually and clearly see the lesion of cervical spinal cord injury but also find that most patients with SCIWORA have tissues compressing the cervical spinal cord, among which cervical disc herniation and ossification of the posterior longitudinal ligament are the most common ones [16, 17]. The persistent compressed tissue aggravates the cervical spinal cord lesion and aggravates the cervical spinal cord dysfunction. Therefore, early surgical treatment is very important.

The results of this study showed that the postoperative JOA score of the observation group was (14.98 ± 2.75) higher than that of the control group (12.16 ± 2.54), and the improvement rate of the excellent and good JOA score in the observation group was also higher than that of the control group. These results indicate that anterior cervical surgery has a good effect on the treatment of SCIWORA and can effectively improve the cervical spinal cord function. The reason was analyzed that conservative treatment with detumescence, inhibition of inflammatory reaction, nerve protection, and other measures to reduce the symptoms of spinal cord compression and improve the protection of the spinal cord in patients but could not quickly relieve the spinal cord compression in patients [18, 19]. Surgical treatment can quickly relieve the symptoms of spinal cord compression, rebuild the stability of the cervical spine, restore the physiological curvature of the cervical spine, and promote the rapid recovery of the spinal cord function of the patient, thereby improving the cervical spine function and neurological recovery. The results of this study also show that after operation, the scores of health condition, physiological function, and role physical in the observation group were (23.18 ± 1.09), (22.75 ± 1.54), and (22.64 ± 1.46), which were higher than those in the control group (20.94 ± 1.65), (20.26 ± 1.78), and (19.56 ± 1.82). These results indicate that anterior cervical surgery for SCIWORA can effectively improve the quality of life of patients.

Univariate and multivariate analysis in this study showed that the ASIA classification of cervical cord injury, the type of MRI cervical cord injury, the scope of cervical cord injury, and the time from injury to treatment were the independent factors influencing the prognosis of patients. The reason is analyzed that MRI can not only visually display different signal changes of the injured spinal cord but also clarify the stage and scope of injury [20, 21]. When the spinal cord injury is milder, the MRI signals are mostly unchanged. The spinal cord injury is more severe, and local blood circulation is impaired, resulting in local edema. With the aggravation of ischemia and hypoxia, local necrosis and cystic degeneration of the spinal cord occur. Spinal cord edema or hematoma after injury causes effective blood circulation disorder of the spinal cord, further aggravates the degree of spinal cord injury in patients, and greatly increases the difficulty of prognosis and recovery for patients. The external force during injury and the compression time of the spinal cord are important factors affecting the neurological recovery after cervical spinal cord injury. Therefore, prompt treatment is extremely important for patients with SCIWORA, and early removal of spinal cord compression and restoration of spine morphology and blood supply are conducive to promoting the recovery of neurological function.

## 5. Conclusion

For patients with SCIWORA, anterior total lamina decompression and internal fixation with bone grafting and fusion can effectively promote the recovery of cervical spinal cord function and improve the prognosis and quality of life of patients. The ASIA classification of cervical spinal cord injury, the type of MRI cervical spinal cord injury, the scope of cervical spinal cord injury, and the time from injury to treatment were the independent prognostic factors for patients.

## Figures and Tables

**Figure 1:** Comparison of the cervical spinal cord function. Note. Compared with before surgery, ^*∗*^*P* < 0.05. Compared with the control group, ^#^*P* < 0.05.

**Figure 2:** Comparison of the curative effect. Note. Compared with the control group, ^*∗*^*P* < 0.05.

**Figure 3:** Comparison of the quality of life. Note. Compared with the control group, ^*∗*^*P* < 0.05.

**Table 1:** Comparison of general data between the two groups.

Group	Age (years)	Gender		Cause of injury		
		Male	Female	Mild	Moderate	Severe
Control group	51.25 ± 9.06	20	18	19	12	7
Observation group	52.04 ± 8.92	29	19	23	16	9
*t*/*X*^2^	0.405	0.524		0.041		
*P*	0.687	0.469		0.981		

**Table 2:** Univariate analysis of prognosis of patients.

Influencing factor	*n*	Excellent group (*n* = 68)	Poor group (*n* = 18)	*X * ^2^	*P*
Gender				1.459	0.227
Man	49	41 (60.29)	8 (44.44)		
Woman	37	27 (39.71)	10 (55.56)		
Age				0.366	0.545
≥50 years	52	40 (58.82)	12 (66.67)		
<50 years old	34	28 (41.18)	6 (33.33)		
Cause of injury				0.902	0.637
Mild external force	42	35 (51.47)	7 (38.89)		
Moderate external force	28	21 (30.88)	7 (38.89)		
Severe external force	16	12 (17.65)	4 (22.23)		
ASIA classification of cervical spinal cord injury				12.006	0.007
Grade *A*	6	2 (2.94)	4 (22.22)		
Grade *B*	18	12 (17.65)	6 (33.33)		
Grade *C*	24	20 (29.41)	4 (22.22)		
Grade *D*	38	34 (50.00)	4 (22.22)		
Types of MRI cervical spinal cord injury				9.784	0.008
No change	30	27 (39.71)	3 (16.67)		
Spinal cord edema	50	39 (57.35)	11 (61.11)		
Intramedullary hemorrhage	6	2 (2.94)	4 (22.22)		
Range of cervical spinal cord injury				12.844	0.002
≤1.5 cm	24	22 (32.35)	2 (11.11)		
1.5∼4.0 cm	57	45 (66.18)	12 (66.67)		
>4.0 cm	5	1 (1.47)	4 (22.22)		
Herniated disk				3.996	0.046
Yes	64	49 (72.06)	17 (94.44)		
No	22	19 (27.94)	1 (5.56)		
Injury to treatment time				10.667	0.005
<3 h	52	43 (63.24)	9 (50.00)		
3∼8 h	24	21 (30.88)	3 (16.67)		
>8 h	10	4 (5.88)	6 (33.33)		

**Table 3:** Multifactor analysis assignment table.

Factors	Variable	Assignment
ASIA classification of cervical spinal cord injury	*X*1	Grade *D* = 0, grade C = 1, grade *B* = 2, grade *A* = 3
Types of MRI cervical spinal cord injury	*X*2	No change = 0, spinal cord edema = 1, intramedullary hemorrhage = 2
Range of cervical spinal cord injury	*X*3	≤1.5 cm = 0, 1.5∼4.0 cm = 1, >4.0 cm = 2
Herniated disk	*X*4	No = 0, yes = 1
Injury to treatment time	*X*5	<3 h = 0, 3∼8 h = 1, >8 h = 2

**Table 4:** Multivariate analysis of prognosis of patients.

Variables	*B*	S.E	Walds	*P*	OR	95% CI
ASIA classification of cervical spinal cord injury	0.392	1.385	4.872	0.038	1.466	1.084∼1.956
Types of MRI cervical spinal cord injury	0.644	0.162	7.968	<0.001	1.946	1.425∼2.683
Range of cervical spinal cord injury	1.305	0.374	8.964	<0.001	2.168	1.596∼2.792
Herniated disk	2.894	3.082	0.386	0.865	18.945	0.071∼58.362
Injury to treatment time	1.132	0.369	9.472	<0.001	3.049	1.614∼5.495

## Data Availability

The datasets used in this study are available from the corresponding author upon reasonable request.
